The article "Assembly operation productivity improvement for garment production industry through the integration of lean and work-study, a case study on Bahir Dar textile share company in garment, Bahir Dar, Ethiopia" was retracted in 2025. Reason: concerns about the citations.

# Assembly operation productivity improvement for garment production industry through the integration of lean and work-study, a case study on Bahir Dar textile share company in garment, Bahir Dar, Ethiopia

**DOI:** 10.1016/j.heliyon.2023.e17917

**Published:** 2023-07-07

**Authors:** Mequanent Ewnetu, Yewondwosen Gzate

**Affiliations:** a Industrial Engineering Department, Institute of Technology, University of Gondar, P. Box.196, Gondar, Ethiopia; b Mechanical Engineering Department, Institute of Technology, University of Gondar, P. Box.196, Gondar, Ethiopia

**Keywords:** Productivity, Lean manufacturing, Work-study, Line balancing, Waste

## Abstract

Productivity improvement is a significant issue for the textile and garment industry to survive global competition. Therefore, the nation's efforts towards this improvement are one of the key weapons to attain cost, time, and quality advantages for rivalry. Ethiopian garment industries are not competitive due to low productivity, which is caused by multidimensional productivity factors related to humans, methods, control, processes, and products. Hence, a single tool or simple model cannot boost significant change for productivity improvement and cannot solve both internal and external productivity factors of the garment industry at this time. However, combined techniques or tools of lean and work-study are preferable. Lean manufacturing is a procedure to identify and eliminate non-value-adding activities in a consistent, continuous improvement. Lean techniques provide a good overview of the processes, whereas work-study methods focus on the critical areas of the operation. This research deals with productivity improvement in the assembly operation of the garment industry with a case study using integrated techniques and tools, such as line balancing, work standardization, time and method study, total working method, and process improvement related to kaizen and 5S. These tools help to eliminate non-value-adding activities were reduce lead time, and defects. The study illustrates, using a case study, the most critical factors that hinder the productivity of Ethiopian garment industries and how to solve these factors through integrated techniques or tools. The research is practical and realistic, and the necessary data was collected using primary and secondary data from the Minister of the Ethiopian garment industry and the case garment. The observed results indicated that non-value-adding activities were minimized from 43% to 5%, bottlenecks from 3 to 0, and the transportation distance of the workers was reduced by 650 m per shift. The daily production output of the case garment and main exports of Flat sheet and Quilt cover products increased from 43.3% to 57.7%–75.8% and 100% pcs per shift, respectively. The standard time for each operator can be set using time study, which can save 315 min for the case garment operation, achieving its production targets of 800 pcs per shift. Therefore, using a single tool or model has not significantly improved this garment industry, but it should be used as a combined tool of lean and work-study for attractive productivity improvement.

The article "Assembly operation productivity improvement for garment production industry through the integration of lean and work-study, a case study on Bahir Dar textile share company in garment, Bahir Dar, Ethiopia" was retracted in 2025. Reason: concerns about the citations.

## 1 Introduction

In the present-day business scenario, every manufacturing (mfg) industry faces increasing competition and hence efforts to be low-cost producers of their products with high productivity [1]. This economic competition is increasing between developed and developing countries [2]. But, the main determinants of the manufacturing firms are no longer the relative cost advantage. Moreover, which based on quality, speed, supervision, and product variation [3]. In the manufacturing industry, whether at the international, national, or firm level, raising productivity is a chief determinant of competitiveness in the global market [2,3]. Because productivity is a measure of the production process, and it reflects the efficiency of the production. Reducing all waste in the mfg. industry can increase production output with a given quantity of inputs [4].

Nowadays, Garment is one of the three basic needs of human beings [5]. Hence, textile and garment manufacturing has retained an important place in human life from the historical era to today's modern world & one of the chief consumer goods [6]. Thus, this sector's production is very intensive [7]. In developing countries, garment industries are more rigorous in sourcing raw materials and minimizing delivery costs than labor productivity because of the availability of cheap labor [8]. The modern garment industry in Ethiopia started in 1958. During- 2019/20, more than 110 textile and 90 garment industries existed in Ethiopia. Entirely it creates job opportunities only for 96,120 workers, which is 47% of the GTP-II plan achieved [9]. The government of Ethiopia has a planned projection of getting 1 billion USD from the export of garment & textile products in 2020 [10]. But, still, now the performance of the Ethiopian textile and garment exports was only $347 million, simply 34.7% achieved, which is much below what the government had planned. The efficiency of this sector during GTPs is slow at 40–45% in production. And average production capacity utilization of this industry at the end of the GTP-II plan-is expected to reach 80%, but now it is below 58% [11]. Nevertheless, Ethiopian garment industries experience growing pressure to improve quality & productivity, reduce cycle time, eliminate errors, improve customer satisfaction, and reduce cost.

The article "Assembly operation productivity improvement for garment production industry through the integration of lean and work-study, a case study on Bahir Dar textile share company in garment, Bahir Dar, Ethiopia" was retracted in 2025. Reason: concerns about the citations.

However, the Ethiopian garment industry and the case of garment are not competitive in the global marketplace because of low productivity and several productivity factors present. These factors are grouped-as human, method, control, process, and product, which require an organized and sustainable productivity improvement program [12]. And the main problems of this garment industry are production under capacity, long lead time, low-skill workers, poor work culture, old machines, low managerial capability, poor system integration, low wage, & export price, limited & low-quality inputs, unbalanced workload, idle time of workers, Poor space and resource utilization, unsuitable working method, high defects & rework. Due to these problems, at this time, the case garment's chief export production process cannot run at the actual capacity, which is 800 pieces per shift. But the actual output is below 470 Pieces per shift, which is approximately 59% only to be achieved [13]. Consequently, this paper aims to improve the productivity of the Ethiopian garment industry as well as the case company via the integration of work-study and lean tools. The main objectives of this paper are to address the following closely interrelated issues: first, to investigate those factors that influence the productivity of the case garment and their indicator, second to identify the combination variables of work-study and lean for productivity improvement, third assess the intervention areas for continuous productivity improvement, the last to develop a proposed solution by using the most critical tools of lean and work-study.

In general, to improve garment productivity, many researchers try to use several techniques and tools for continuous productivity improvement separately, but one of each technique doesn't improve productivity comprehensively [12,13]. So, this gap helps this study to find more comprehensive improvement tools & techniques which can solve both internal and external productivity factors, which enhance the overall productivity of the garment industry. These preferable techniques are the integration of lean and work-study. So, using these integrated tools to form an inclusive & reliable set of industrial practices, their synergy is supportive and contributes hopefully to continuous productivity progress [13]. Because-lean tools are commonly used to identify and eliminate eight wastes and create a non-stop perfection in the production flow, while work-study techniques improve workers' processes and eliminate unnecessary time spent on critical work areas [14]. Hence, this study tries to identify & solve these factors by these integrated improvement tools and techniques that enhance a significant change in productivity improvement.

The article "Assembly operation productivity improvement for garment production industry through the integration of lean and work-study, a case study on Bahir Dar textile share company in garment, Bahir Dar, Ethiopia" was retracted in 2025. Reason: concerns about the citations.

This study was limited to productivity improvement for the Ethiopian garment industry, and the case study was conducted only on Bahir Dar Textile Share Company in Garment by identifying the most significant internal & external productivity factors. However, it did not address all productivity factors for each garment industry because of resource & time constraints. Additionally, there was limited access to data due to Covid-19.

### 1.1 Literature review

#### 1.1.1 Concept of productivity

The word productivity is not new and has been used for centuries. Initially, productivity was viewed mainly as an efficiency concept. However, today, productivity measures system performance, system efficiency, resource utilization, and the relationship between actual output & input. The economic growth of any country is usually measured by an increase in production, which comes from two sources: a larger quantity of production factors used (inputs) or an increase in productivity [15]. Therefore, productivity is a component of growth. To minimize the loss of factors related to labor, machines, and material provided to increase productivity. The European Productivity Agency has defined productivity as an attitude of mind. It is a measure of the degree of effectiveness & efficiency of any service and manufacturing organization in generating output, given the resources available. Defining the inputs and outputs is very crucial and mandatory. Nowadays, the inputs of the manufacturing industry include materials, machines, humans, methods, technology, land, building, money, market, management tools, and information.

In general, the inputs of all firms are considered to be human, capital, material, energy, and various miscellaneous inputs. The outputs are finished products, partial products for sale, and internal use. Methods are means applied to do activities efficiently, while control deals with regulating activities and parameters within an acceptable limit. All operation and non-operation times were carefully considered in the operation. Waste is part of the resources that have no purpose or value to the firm and customers [15,16]. Thus, productivity is defined as the effective and efficient utilization of resources used to produce products or services that meet customer wants continuously by applying suitable methods and time through controlling the parameters of constraints that help any industry to survive in a global market share.

#### 1.1.2 Productivity improvement

Since the 1950s, the struggle between companies has increased as markets have become increasingly global. This has created a greater need for first-rate improvement approaches to sustain competitiveness. Improving productivity has a positive impact on the direct costs of products, as the same output is produced with less input or as the same inputs are producing more output [17]. Productivity improvement focuses on doing the “right things” by continuously reviewing and identifying changing customer and societal needs. The rate at which a company produces goods/services is related to the number of materials and the number of employees needed [17,18]. Hence, productivity improvement can be achieved by sorting or elimination, reducing variation, repairing ineffective processes, simplifying the method, optimizing the system, maximizing turnout-up quality or responsiveness, and reducing set-up time [18]. Improving productivity means increasing the efficiency and effectiveness of changing inputs into outputs or the elimination of waste [19]. To achieve continuous productivity improvement, improvement tools that solve all barriers being used in the industry, such as lean, Just-in-time, 5S, standardized work, value stream analysis, Pareto, cause-effect diagram, cost/benefit analysis, continuous flow, Heijunka, Jidoka, etc., are utilized [20]. The two vital functions that help to increase productivity are the installation of the most effective method of operating and the control of resources. This thought addresses the main elements of competition: innovation, cost, quality, and time [20]. In summary, productivity improvement is one of the most vital factors for any textile and garment industry to increase the efficiency and effectiveness of the transformation of input into outputs to survive in this global upward competition. Because globalization has given rise to new standards by increasing the value-added content of products, decreasing the unit cost and work content of production, and line balancing of methods, a combination of all using appropriate techniques, tools, and approaches is necessary.

The article "Assembly operation productivity improvement for garment production industry through the integration of lean and work-study, a case study on Bahir Dar textile share company in garment, Bahir Dar, Ethiopia" was retracted in 2025. Reason: concerns about the citations.

#### 1.1.3 Concept of lean manufacturing

The word “Lean” is a powerful and capable term that also refers to being slim and fit [20]. The concept of Lean was originally developed in Japan by Toyota for their automobile manufacturing, replacing mass production Womack and Jones (1990). Lean manufacturing describes a system that produces what the customer wants, when they want it, with minimum waste. Its concept arises when a company wants to make the process more efficient, without delays, and with less capital and can be used in automobile, garment, aerospace, chemical engineering, or any manufacturing industry [21,22]. Lean manufacturing (LM) is a procedure to eliminate waste reliably through continuous improvement in manufacturing industries [23]. Thus, the idea behind the Lean concept is to maximize customer value while minimizing waste to increase the value of the products [24]. The main objective of Lean manufacturing is to reduce the overall production cost, increase efficiency, and minimize the overall lead time [24].

Lean manufacturing (LM) has a comprehensive set of rules, elements, and tools and focuses on removing waste and creating value. One of the crucial aspects of Lean manufacturing is the never-ending quest for perfection, the continuous search to eliminate waste, and the recognition and importance of employee contributions. Its primary aim is to attain the same output with less input, less time, less space, less human effort, less machinery, less material, and low cost [25]. Hence, Lean manufacturing helps to identify productively value-adding and non-productive non-value-adding activities [26]. At present, Lean production aims to increase productivity, improve product quality, reduce manufacturing cycle time, reduce inventory, reduce lead time, and eliminate manufacturing waste using Lean tools such as Kaizen, Kanban, 5S, JIT, VSM, etc. [27]. The organizational benefit of Lean manufacturing is superior management, reduced waste in human effort, production space, less rework, improved quality, faster delivery time, increased worker efficiency, total involvement, problem elimination, increased space utilization, safer work environment, and improved employee morale [28].

The application of Lean practices can be difficult due to various factors such as the dependence on suppliers due to a small amount of inventory, high cost of carrying out, rejection of employees and poor workplace, focus on waste elimination, and lack of attention to other limits such as workers' safety and ecological risk, which are not considered as waste in Lean manufacturing [27,28]. However, Lean manufacturing is still one of the systematic approaches used to identify and eliminate wastes through continuous improvement, and the production flow at the pull of the customer is in search of perfection in any garment industry for enhancing productivity.

#### 1.1.4 Lean tools

There are over 30 types of Lean tools that can be used to improve manufacturing processes. These tools can be grouped into categories such as process and work method, time, management and control, quality, and human safety, based on their practical use in Lean manufacturing [27,28]. Learning and implementing these tools and techniques can be good industrial engineering practices that can be functional for different companies in many contexts and without difficulties.

The article "Assembly operation productivity improvement for garment production industry through the integration of lean and work-study, a case study on Bahir Dar textile share company in garment, Bahir Dar, Ethiopia" was retracted in 2025. Reason: concerns about the citations.

#### 1.1.5 Wastes of lean manufacturing

In Lean manufacturing, anything that doesn't add value to the manufacturing process is considered waste. This means any procedure for which the customer does not pay the company. Wastes are usually caused by unnecessary delays, processes, costs, and errors [29]. These wastes can be generated due to poor layout, long setup time, incapable processes, poor work methods, lack of training, large batches, ineffective production planning, lack of workplace organization, etc. The wastes (Muda) in Japanese can be categorized into seven forms: defects, waiting, overproduction, conveyance, processing, inventory, and motion. These types of waste have their causes and solutions, and when eliminated, provide multiple benefits [30]. There are eight Lean manufacturing wastes: over-processing, waiting, and unnecessary (motion, transportation, and inventory), over-processing, unused skills, and defects. In general, all these Lean wastes should be reduced or eliminated in any manufacturing industry, such as the textile & garment industries, using these integrated tools to enhance the productivity of the Ethiopian garment industry.

#### 1.1.6 Work-study

Work-study is a vital technique in any industry as it can be implemented with less investment or no investment to enhance production efficiency, reduce costs, and strengthen competitive ability by improving the operating process and method, fully utilizing human, material, and financial resources within the firm [30]. Work-study aims to find the best and most efficient way of utilizing available resources to achieve the best possible quality of work in the minimum possible time and cause the least potential fatigue to the worker. The importance of this technique lies in enhancing production efficiency and identifying non-value-adding operations by examining all the factors that affect the job and setting standards. By using work-study, companies can identify and eliminate waste, improve productivity, and reduce costs. This technique can be applied to various industries, including the textile and garment industries, to improve their production processes and increase their competitiveness in the market.

#### 1.1.7 Purpose of work-study

The main objectives of work-study are to establish the most economical way of doing the work, to determine the time required for a job at a defined level of performance, to increase productivity, profitability, and job security, to make work easier, establish fair tasks for everyone, check achievements against standards, and to install the work method as standard practice [31].

The article "Assembly operation productivity improvement for garment production industry through the integration of lean and work-study, a case study on Bahir Dar textile share company in garment, Bahir Dar, Ethiopia" was retracted in 2025. Reason: concerns about the citations.

#### 1.1.8 Techniques of work-study

Work study is mostly categorized into two techniques: method study and work measurement. Method study focuses on searching for an efficient working method, while work measurement determines the scientific and reasonable working time quota of each operation [32]. See the following Figure.

#### 1.1.9 The relationship between work-study and productivity

Work-study has received necessary acclaim in the clothing industry due to its positive effects on productivity, quality, and competitiveness (see Fig. 1). By using work-study techniques, companies can increase their productivity by identifying and eliminating non-value-adding operations, simplifying tasks, and improving the layout of the workspace. See in Fig. 2. The relation between work-study and productivity.

**Fig. 1:** Work-study techniques [32].

**Fig. 2:** The conceptual model of work-study and productivity [33].

#### 1.1.10 Integration of lean and work-study

Lean manufacturing and work-study are both popular techniques that have been widely used to improve quality and productivity in various industrial sectors, including the garment industry, with high success rates [33]. These techniques are used to reduce waste caused by excess inventory and over-production in the warehouse. Lean manufacturing is implemented with flow process charts to maximize production efficiency [34]. When used together, lean manufacturing and work-study techniques can provide a universal solution for any industry facing productivity challenges. By combining these techniques, companies can improve their performance, and if implemented in the proper order, 100% positive results are assured [35]. Therefore, to implement work-study and associated lean tools in the garment industry, it is important to cover technical, engineering, and manufacturing aspects, as well as business customs affairs. Lean manufacturing has changed the manufacturing environment, requiring work-study to change and develop to meet the requirements of the new manufacturing setting, which focuses on working smarter, not harder [34,35]. Despite the widespread use of lean manufacturing and work-study techniques, there are still questions regarding the gap between their applications. One study aims to address this gap by reviewing various literature sources. It was found that lean manufacturing provides a good overview of the processes, while work-study focuses on critical areas of the operation. Therefore, both techniques are highly effective for improving productivity in any manufacturing industry.

## 2 Methodology

The methodology used as combined techniques or tools of lean and work-study and this research was conducted in the Ethiopian garment industry, specifically in the case garment industry. To achieve the research objectives, a combination of primary and secondary sources, as well as qualitative and quantitative methods, were used to collect relevant data. The data was collected through direct observation, interviews, data recording and measuring, questionnaires, and secondary data methods. The collected data was analyzed and presented using SPSS and Qi-Macro's software, as well as various lean and work-study tools.

The article "Assembly operation productivity improvement for garment production industry through the integration of lean and work-study, a case study on Bahir Dar textile share company in garment, Bahir Dar, Ethiopia" was retracted in 2025. Reason: concerns about the citations.

### 2.1 Data collection and analysis

To collect data and understand the existing productivity factors, improvement approaches, and practices of Ethiopian garment industries, primary data and a literature survey from ETIDI and Bahir Dar Textile Share Company in garment production were conducted. Qualitative data was collected using simple random sampling methods, and a questionnaire was prepared with four major parts. The questionnaire was disseminated to the estimated sample size of 102, and all responses were received without missing variables, meeting the estimated sample size. The qualitative data were analyzed using SPSS-V 21 software, and data validation was checked using the SPSS case process summary table to read the values of the Chi-Square, Hosmer, and Leme show test. The data was found to be valid, and the analysis showed that most of the estimated variables that were drawn in the regression were fit, with values (p values) less than 5%.

### 2.2 Frequency distribution for eight wastes of (lean) of the respondents

According to the respondents' responses, the most frequently occurring lean wastes in the case garment were input defects (63.7%), unnecessary motion (61.7%), waiting (64.7%), and excessive transportation (65.7%). These wastes were identified as one of the main factors contributing to the low productivity of the case garment. Fig. 3 shows the frequency distribution of lean wastes, with the coding “No” indicating that the wastes did not occur frequently, indicating that the company was productive. On the other hand, the coding “Yes” indicates that these wastes occurred repeatedly, leading to low productivity in the case garment. It was found that over-production and inventory were not productivity factors for this company.

**Fig. 3:** Frequency distribution of lean wastes in the case of the garment.

## 3 Result and discussion

### 3.1 Qualitative data analysis by multivariate logistic regression analysis

Multivariate regression was used to regress several dependent variables jointly with the same independent variables to identify the most critical productivity factors associated with low productivity in the case company (see Table 1). This regression is a joint estimator between equation covariance and can be tested coefficients across equations. The multivariate logistic regression was analyzed using entering, forward, and backward-conditional methods and the result of this analysis had the same values. The data validation test of this regression was taken in 9 iterations, and the result indicates that the ten most critical productivity factor variables were found from these internal, external, and waste factors. These include low-quality inputs (COR = 0.338 and AOR = 0.116), poor working method (COR = 0.206 and AOR = 0.059), long lead time (COR = 0.161 and AOR = 0.258), etc. (see Table 2). The multivariate regression analysis was found to be fit, and the collected data was valid in the model when the significance level (*P*-value) was greater than 5%, and the values of the Chi-square test were below 5% (Hosmer and Leme show estimation). The summarized table is provided below.

The article "Assembly operation productivity improvement for garment production industry through the integration of lean and work-study, a case study on Bahir Dar textile share company in garment, Bahir Dar, Ethiopia" was retracted in 2025. Reason: concerns about the citations.

**Table 1:** The most commonly known lean tool and techniques [28].

Lean tools and techniques		
5S	Jidoka- Automation	Multi-function employees
VSM	Muda (waste)	Root cause Analysis
Cell Layout	PDCA (plan-Do-Check and Act)	Single piece flow
Kaizen	Standardize work	Team Building
Poka-Yoke (error-proofing)	Bottleneck analysis/line balancing	Gemba
JIT	Kanban (pull system)	Visual display & control
TPM	Heijunka - level scheduling	Supplier management
Single-Minute Exchange of Dies	Visual Management	Small lot size
Cellular manufacturing	Flow production	Uniform workload

**Table 2:** Multivariate logistic regression of the most critical productivity factors.

The most critical factors	Level	*P*- Value	AOR	95% C.I. for Exp (B)	
				Lower	Upper
Limited and low-quality inputs	0. No 1.Yes	.016	.116	.020	.667
Inappropriate working method & process flow	0. No 1.Yes	.009	.059	.007	.496
Long lead time	0. No 1.Yes	.012	.258	.051	1.31
Less export price of the product	0. No 1.Yes	.023	.131	.023	.751
Unbalanced workload between workers	0. No 1.Yes	.018	.092	.013	.666
Poor infrastructure & utility center	0. No 1.Yes	.002	.044	.006	.314
Human resources & dept. center	0. No 1.Yes	.010	.162	.040	.651
Quality control department	0. No 1.Yes	.000	.061	.013	.286
Waiting time	0. No 1.Yes	.018	.363	.156	.843
Defects	0. No 1.Yes	.003	.052	.008	.753

To summarize, the data was found to be valid, and the most critical productivity factors were identified in the garment industry through a literature review and an overview of Ethiopian garment industries. Qualitative data analysis was used to identify the most critical productivity factors of the case garment, and this will help in the detailed investigation of these factors using quantitative data methods.

The article "Assembly operation productivity improvement for garment production industry through the integration of lean and work-study, a case study on Bahir Dar textile share company in garment, Bahir Dar, Ethiopia" was retracted in 2025. Reason: concerns about the citations.

### 3.2 Quantitative data analysis by the existing working method flows and waste analysis

The study primarily focused on examining the most critical internal productivity factors, such as excessive motion, working method, long-lead time, and ineffective resource utilization. These factors lead to the tasks faced for many discrete activities, and the movements of materials and operators going over a long distance between each operation. This creates a bottleneck between each activity, holding up other production processes, which are lengthy and consume a long time. Fig. 4 provides a visual representation of this issue.

**Fig. 4:** The existing working methods with its detailed activity flow of the case garment.

Fig. 4 illustrates the long path of movements required to complete production operations, as measured by distance traveled and time. This results in improper line balancing and an irregular sequence of activities, leading to slow input material and product feeding to the machine. The spreading cutting machine, which is at the center of garment production, creates a bottleneck, causing high lead time, material handling cost, backtracking, hazards to personnel, less labor efficiency, minimized employee morale, and decreased daily production output. To address this issue, the castoff method study technique was used to critically examine the current method by observing, measuring, and recording the case garment's detailed activities. Material-type flow process charts were analyzed using descriptive control charts, which show the mean, standard deviation, and range. An X-bar chart was used to monitor the change in the mean of a process or central tendency [16].

(1) $$Mean\;can\;measure\;central\;tendency;\;\bar{x}=\frac{\sum_{i=1}^{n}x_{i}}{n}$$

Where $x_{i}=number\;of\;activities$ [10,16].

(2) $$Range\;\left(r\right)=1_{\max}^{st}-2_{\min}^{nd}$$

(3) $$Standard\;deviation\;\left(\sigma \right)=\sqrt{\frac{\sum_{i=1}^{n}{\left(x_{i}-\bar{x}\right)}^{2}}{n-1}}$$

So, calculate the upper control limit, control limit, and lower control limit by three Sigmas.$UCL=X+Z\sigma_{\bar{X}}\text{;}$ Where zis3sigma,CL=X.

$$LCL=X-Z\sigma_{\bar{X}},\sigma_{\bar{X}}=\frac{\sigma }{\sqrt{n}}$$

Fig. 5 highlights the presence of high non-value-adding activities in the case garment. Poor work methods were identified as one of the main reasons for the high non-value-adding operations, leading to long-distance travel, tightness, backtracking, increased scrap rate, and bottleneck in production. These issues resulted in low productivity, worker fatigue, and stress. The chart also shows the total production operations process, with 12, 9, and 4 activities in control, out of control, and under low control limits, respectively. The next step is to calculate the upper control limit, control limit, and lower control limits to determine whether the process activities are under control or not [10]. (see Fig. 6)

(4) $$Value-adding\;ratio=\frac{Non-Value\;adding\;activities}{Value-adding\;activities}$$

Non−Value−addingactivities=Leadtime−Valueaddingactivities

**Fig. 5:** The SPC chart of the current distance for the case garment production.

The article "Assembly operation productivity improvement for garment production industry through the integration of lean and work-study, a case study on Bahir Dar textile share company in garment, Bahir Dar, Ethiopia" was retracted in 2025. Reason: concerns about the citations.

**Fig. 6:** The existing revised distance for value & non-value-add activities chart [34].

The chart shows, about 43% of the activities are out of control, indicating excessive distance traveled in each production process. To eliminate non-value-adding activities, it is essential to consider different requirements such as space, machines, the number of operators' availability, and so on. By doing so, the production process can be optimized to reduce non-value-adding activities, improve productivity, and reduce worker fatigue and stress.

After the fifth iteration, most activities are under the control limit, and the production process becomes smoother. However, it is still important to address the activities that are out of control to ensure that the production process is optimized and all activities are value-adding for the case garment. By continuously monitoring and improving the production process, the company can achieve higher productivity, reduce waste, and improve the overall quality of the product (see Fig. 7).

### 3.3 A proposed solution for working method, flow, and waste analysis

By using integrated techniques such as 5S, standardized work, SMED, and method study, the company can develop a practical, economical, and effective method for improving the production process and increasing export production volumes. By eliminating non-value-adding activities, combining some parts, and changing the sequences of existing methods, the proposed working method can be optimized to meet customer requirements and improve overall productivity. It is important to consider different improvement alternatives and select the best improvement working method from start to end in the case of garment production, as shown in Fig. 8.

**Fig. 7:** The third revised activity distance iteration chart [35].

**Fig. 8:** The proposed production process of the case garment.

**Fig. 9:** The proposed distance and value-adding activity chart of the case garment [35].

The following Table clearly shows the detailed flow process chart of the case garment production operation.

The company has made progress in eliminating non-value-adding activities and developing a new production flow (see Fig. 9). However, as shown in Table 3, there is still room for improvement in terms of reducing the distance of the production line and reducing the operation time for each activity. By reducing the distance of the production line and optimizing the operation time, the company can further improve productivity and reduce waste. The proposed changes can be seen in the following Figure.

The article "Assembly operation productivity improvement for garment production industry through the integration of lean and work-study, a case study on Bahir Dar textile share company in garment, Bahir Dar, Ethiopia" was retracted in 2025. Reason: concerns about the citations.

**Table 3:** The proposed material flow process chart of the case garment industry.

As shown in the chart, the percentage of value-adding activities has increased from 57% to 95%, which is a significant improvement (see Fig. 10). While there are still a few activities that cannot be eliminated, they can be minimized and considered as value-adding activities. The comparison between the existing and improved working methods in Fig. 11 shows that most of the existing production wastes or problems have been solved. Overall, the company has made great strides in improving the garment production process and increasing productivity.

**Fig. 10:** Chart showing adding and non-value-adding activities [34].

**Fig. 11:** The comparison between the existing and improved production flow activity chart.

In summary, Fig. 11 illustrates a significant improvement in the garment production process. The existing process had high movement and non-value-adding activities, particularly for long distances (9 activities = 43%), with only 12 activities (57%) being value-adding. However, after the improvement, the total distance was reduced from 131.8 m to 99.3 m, with an average of 20 movements per operator per shift. This translates to a saving of 650 m per shift. Additionally, non-value-adding activities decreased from 43% to 5%, and bottlenecks were eliminated from 3 to 0. The actual daily output for Flat sheet production was 43.3% per shift, but after the improvement, it increased to 75.8%. To achieve the production target of 800 pieces per shift in the garment case, the focus was primarily on reducing production time. Therefore, it is crucial to maintain a new method to monitor the effectiveness of the improved working methods and personnel's adaptation. Sometimes, the effect of the new work method on other activities is overlooked. For instance, the new work method successfully eliminated the bottleneck in a particular area of the production process. By periodically checking the proposed working method and its effects, the management can ensure that overall efficiency is improving rather than deteriorating. The main focus of this study was to conduct a detailed investigation of the problems in the garment industry that can be solved based on actual data. This involved the direct recording and measuring of facts while considering industry standards.

The article "Assembly operation productivity improvement for garment production industry through the integration of lean and work-study, a case study on Bahir Dar textile share company in garment, Bahir Dar, Ethiopia" was retracted in 2025. Reason: concerns about the citations.

## 4 Conclusion

Improving productivity through the integration of lean and work-study tools is a crucial issue in the textile and garment industry. This approach is practical and cost-effective for enhancing productivity. While the garment industry is a basic human need, it faces multidimensional productivity factors that do not have an equal effect on each garment industry, including the case of the garment. Therefore, this investigation focused on identifying the critical productivity problems in garment production and solving them using line balancing, work standardization, time and method study, and total working method and process improvement related to kaizen and 5S. The study used reliable data to identify the most critical internal, external, and lean waste productivity factors and assessed the correlation and regression between the dependent variable (productivity) and independent variables (all factors). The analysis indicated a strong correlation and significance value between them.

The values of ‘r' (0.75) and p-value (below 5%) indicate a strong correlation and significance between the dependent variable (productivity) and independent variables (all factors). The overall finding of this study suggests that reducing non-value-adding activities such as unnecessary motion, waiting time, production flow, and transportation, as well as reducing bottlenecks, backtracking, and production costs, while increasing the utilization of workers, machines, and space, can create the best working method and process and increase operator efficiency. Based on the analysis, the following results were obtained: non-value-adding activities can be reduced from 43% to 5%; bottlenecks can be reduced from 3 to 0; and creating better working methods and flows can reduce the total garment operation activity distance to 650 m per shift per day. The actual daily output in percent for Flat sheet and Quilt cover products is 43.3% and 57.7% pieces per shift, respectively. However, after improvement, it can be increased to 75.8% and 100% pieces per shift, respectively, and standard time and daily outputs can be set for each operator. As a result, the company can save 315 min for this production operation, achieving their production targets of 800 pieces per shift. This improvement eliminated the need for an additional shift to achieve the targets, which was required before studying this research. It also helped to reduce the high production costs that the company was inquiring about before the improvement. In conclusion, implementing these integrated techniques can lead to continuous productivity improvement in the Ethiopian garment industry, as demonstrated by the case of garment where all productivity factors were solved using these techniques. However, it is important to note that overall productivity improvement in the garment industry cannot be achieved using a single tool or developing a simple model.

The article "Assembly operation productivity improvement for garment production industry through the integration of lean and work-study, a case study on Bahir Dar textile share company in garment, Bahir Dar, Ethiopia" was retracted in 2025. Reason: concerns about the citations.

### 4.1 Future research work

The Ethiopian service and manufacturing industries are the main economic drivers of the nation. Future research in this area should focus on using these integrated techniques to develop appropriate methods that improve productivity in the garment industry. While this study specifically focused on Bahir Dar Textile Share Company in the garment industry, it would be beneficial to implement these techniques and assess their impact on other Ethiopian garment industries. Additionally, a detailed investigation of ergonomics assessment in all Ethiopian garment industries, including the case garment, is needed. Finally, designing a conveyor belt system to transport garment products/materials in the sewing operation process could also be explored as a potential solution to improve productivity in the industry.

## Author contribution statement

Mequanent Ewnetu: Conceived and designed the analysis; Analyzed and interpreted the data; Contributed analysis tools or data; Wrote the paper.

Yewondwosen Gzate: Contributed analysis tools or data; Wrote the paper.

## Data availability statement

Data included in article/supp. material/referenced in article.

## Declaration of competing interest

The authors do not declare any competing or non-financial interest.
